# Effective role of lady health workers in immunization of children in Pakistan

This article has been retracted.

**DOI:** 10.12669/pjms.326.11460

**Published:** 2016

**Authors:** Saira Afzal, Azka Naeem, Unaiza Shahid, Wajiha Noor Syed, Urva Khan, Nayyar Misal Zaidi

**Affiliations:** 1 Dr. Saira Afzal, MBBS, MPhil, MCPS, FCPS, PhD Post Doctoral Fellow (US), Chairperson and Head, Department of Community Medicine, Faculty of Public Health, King Edward Medical University, Lahore, Pakistan; 2 Azka Naeem (MBBS Student KEMU), King Edward Medical University, Lahore, Pakistan; 3 Unaiza Shahid (MBBS Student KEMU), King Edward Medical University, Lahore, Pakistan; 4 Wajiha Noor Syed (MBBS student KEMU), King Edward Medical University, Lahore, Pakistan; 5 Urva Khan (UK Student KEMU), King Edward Medical University, Lahore, Pakistan; 6 Nayyar Misal Zaidi (MBBS Student KEMU), King Edward Medical University, Lahore, Pakistan

**Keywords:** Lady health worker program, Immunization, Determinants

## Abstract

**Objective:**

To determine the association of Lady Health Worker’s role with immunization of children in Pakistan.

**Methods:**

Secondary analysis was conducted on data obtained from Pakistan’s Demographic and Health Survey. Children who did not receive all doses of vaccines were considered incompletely immunized or vice versa. The association between determinants was assessed by simple and multivariable binary logistic regression.

**Results:**

The mothers and fathers had a mean age of 32.7 (SD+8.6) years and 37.9 (SD +10.1) years, respectively. Age of mother greater than 35 (OR=0.93; 95% CI:0.70-1.25); born in Baluchistan (OR=3.47,95% CI:2.21-5.49); rural area dwellers (OR=2.04; 95% CI:1.65-2.51); female gender (OR=1.06; 95% CI:0.87-1.29); birth order (of last born child) greater than 7 (OR=2.21, 95% CI:1.60-3.06); delivered at home (OR=2.20, 95% CI:1.76-2.74); long distance to health care facility (OR=2.66, 95% CI:2.16-3.28); and no LHW visit in last 12 months (OR=1.91, CI:1.48-2.47) were significantly associated with incomplete immunization in bivariate analysis. In final model of multinomial regression analysis the absence of visit by LHW in last 12 months was the most significant factor when all risk factors were analyzed in last model

**Conclusions:**

This study has concluded that visit of LHW in last 12 months was significantly associated with immunization.

## INTRODUCTION

According to the World Health Organization (WHO), the past decade was supposed to be “a decade of vaccines.”^1^ The goal, however, has yet to be fully accomplished. Universally, WHO efforts have reduced the global burden of under-five deaths from 12 million to 6.6 million. Despite this progress, Pakistan ranked 26 internationally for under-five mortalities, with an under-five mortality rate of 86 per thousand live births. Furthermore, Pakistan has a neonatal mortality rate of 42 per thousand live births, and an infant mortality rate of 69 per thousand live births.^1^ In response to this health need, WHO introduced the Expanded Program of Immunization to address the leading cause of these mortalities, vaccine-preventable diseases, and to ultimately achieve the Millennium Development Goal 4 (reduce child mortality).^2^ Despite the universal acceptance of this program, equal distribution of immunization rates has still not been achieved globally. Potential causes include lack of community awareness and participation, inaccessibility of health facilities, and social problems.

To tackle all these problems, the government of Pakistan launched the Lady Health Workers program in conservative rural and under-developed communities. Conservative communities didn’t allow the strangers and outsiders to interact with their women and children. A study in Pakistan in 2007 stated that 66% of children were incompletely immunized due to birth at home, demonstrating the need for active community outreach.^3^ The program workers deliver door-to-door preventive and curative services to vulnerable communities. In response to the program, 60% of the total rural population of Pakistan covered by the LHW program showed significantly better health indicators.^4^ Furthermore, a randomized control trial conducted in seven subdistricts of Pakistan in 2005 showed that intervention groups receiving health facilities by LHWs showed lesser perinatal and maternal deaths.^5^ Similarly, a survey conducted by United States Agency for International Development (USAID) in November 2012 demonstrated that LHWs increased coverage of fully immunized children among poorer households.^6^

Despite its initial success, LHW program eventually faced challenges and struggled to meet targeted immunization rates. A survey conducted in Karachi in 2008 revealed the LHW program was plagued by lack of incentives, restricted mobility of health workers, lack of interest of doctors and staff, flaws in monitoring of regular vaccination and job dissatisfaction.^7^ A cross-sectional study conducted in Rawalpindi 2008 described low pay, long travel distances, inconsistent medical supplies, inadequate stipends and lack of career structure as common causes of job dissatisfaction among LHWs.^8^

As majority of Pakistan’s population is of rural dwellers, we need to augment and promote the Lady Health worker program, LHWs perform vital roles in immunization campaigns such as the Polio Eradication Initiative and Supplemental Immunization Activities. Hence, this study to emphasizes the indispensable role of LHWs incomplete immunization coverage of children and critically analyzes the problems encountered in implementation of LHW program.

## METHODS

We conducted secondary analyses of data from Pakistan Demographic Survey (PDHS) 2012-13. PDHS is a cross-sectional survey, funded by USAID. The survey was done to have unbiased information on health-related variables including immunization, maternal and child health, nutritional status of mothers and children, and awareness regarding communicable diseases. It is considered as a nationally representative survey providing estimates free of systematic bias. It was designed to include 13,944 households; however, the final sample size consisted of 12,943 households (96% response rate). The details of methodology of the survey can be accessed elsewhere.^9^

We restricted our research mainly to variables related to child immunization. Our data was limited to mothers with her youngest child between the ages of 12 to 23 months, resulting in a samples size of 3,294. The reason of the selection of this age group was that the course of basic vaccinations (i.e., 12 doses for seven vaccine-preventable disease i.e. VPDs) for children is completed by the age of 9 months, with booster dose of Measles vaccination at the age of 15 months. Secondly, previous studies have also used the same age-group to assess the immunization status of children.^10^-^12^

The dependent variable, “immunization status” was computed by using twelve doses of 5 vaccines (i.e. polio (4 doses), BCG (1 dose), DPT (3 doses), HBV (3 doses) and measles (1 dose)). We selected twelve variables, BCG, polio (0,1,2,3), DPT (1,2,3), HBV (1,2,3) and measles. These variables each had four response categories: No vaccination date on card, reported by mother, vaccination marked on card and don’t know (DK). Each variable was coded. No vaccination on card and DK responses were recoded as “0” and considered as “not received the vaccine”, while the other responses “vaccination date on card, reported by mother” were recorded as “I” and considered as “received the vaccine”. Later, we considered all twelve vaccine variables and assigned each child an “Immunization status”. The immunization status was recorded as: “I” for “complete immunization” and “0” for “incomplete immunization”. “Complete immunization” was defined having received one dose of BCG vaccine against tuberculosis; three doses of DPT vaccine to prevent diphtheria, Pertussis, and tetanus (DPT); at least three doses of polio vaccine; and one dose of measles vaccine. “Incomplete immunization” was defined as having missed any or all doses of vaccines. This categorization method was designed along previous research studies definitions.^13^-^15^

The independent variables used in our study were established on an extensive literature review,^13^-^15^ They included: mother’s age, father’s age, mother’s education, father’s education, father’s occupation, wealth index, sex of child, birth order of child, single or multiple gestation, place of residence, years since first cohabitation, access to information, use of antenatal care, place of delivery, respondent’s visit to health care facility in last 12 months and distance of health care facility.

### Statistical Analysis

The data was analyzed by Statistical Package for Social Scientists version 21. Descriptive statistics of children with complete and incomplete immunization were presented as frequency distributions and percentages.

The relationship between all independent variables and outcome of interest (i.e. incomplete immunization) was computed by simple binary logistic regression. The odds ratios, p-values and 95% confidence intervals calculated for association between dependent variable and each independent variable.

The logistic regression was used to assess the relationship between immunization status and visit of LHW in last 12 months. In model one, multiple multinomial logistic regressions were carried out to adjust for different independent variables. In models two and three, the associations of interest were assessed by adjusting for demographic variables of the mother and father (age, education and wealth index), respectively. The relationship was also assessed in model 4 by adjusting for place of residence and region. In model 5, we adjusted for the independent variables related to child (Birth Order, gender and multi-gestation). All the maternal-related independent variables were adjusted in the model 6 (place of delivery and health care facility). Model 7, our final model, evaluated the association of interest by including all the independent variables. We also assessed the multicollinearity between the variables and highly correlated variables were eliminated from the final model. Multicollinearity was assessed between mother’s age and between wealth index and residence, through Pearson correlation, and it was significant at the 0.01 level, so the variables of father’s age and residence were eliminated from the final model. All the analyses were done by using sample weights to produce nationally representative estimates.

## RESULTS

The mothers and fathers had a mean age of 32.7 (SD+8.6) years and 37.9 (SD +10.1) years, respectively. The number of incompletely immunized children increased as the education of the parents decreased. Children were more likely to be incompletely immunized if father’s age was 35 years or more and occupation was manual worker (49%). Children with higher birth order (7 or more), female child (51%), rural place of residence (74.9%) and those belong to low (poor) wealth index (53.9%) were incompletely immunized. (Table-I)

**Table-I:** Frequency distribution and percentages of study variables.

S.	Variables	Participants		

		Incomplete immunization N (weighted%)	Complete immunization N (weig1hted%)	Total
1.	Mother’s age (years)			
	>35	420[20.7]	217[18.7]	637[20]
	25-34	1135[56]	683[58.8]	1818[57]
	15-24	741[23.3]	261[22.5]	3188[23]
	Total	2027[100]	1161[100]	3188
2.	Father’s Age (years)			
	>35	943[47.2]	547[47.5]	1490[47]
	25-34	921[46.1]	539[46.8]	1460[46]
	15-24	134[6.7]	65[5.7]	200[7]
	Total	1998[100]	1152[100]	3151
3.	Mother’s Education			
	Higher Level	127[6.3]	176[15.2]	303 [10]
	Up to Secondary Level	277[13.7]	326[28.1]	604[19]
	Up to Primary Level	328[16.2]	190[16.4]	519[16]
	No education	1293[63.8]	467[40.3]	1761[55]
	Total	2027[100]	1161[100]	3188
4.	Father’s Education			
	Higher Level	264[13.1]	265[23.0]	530[17]
	Up to Secondary Level	629[31.2]	459[39.6]	1088[34]
	Up to Primary Level	320[16.0]	166[14.4]	486[15]
	No education	800[39.7]	266[23.0]	1067[34]
	Total	2016[100]	1158[100]	3174
5.	Father’s Occupation			
	Management/Professional	121[6.0]	133[11.5]	255[8]
	Clerical/Sales/Service	469[23.2]	305[26.3]	774[24]
	Manual worker	993[49.0]	591[51.0]	1584[50]
	Agriculture	399[19.7]	121[10.4]	521[16]
	Not working	42[2.1]	9[0.8]	51[2]
	Total	2027[100]	1160[100]	3188
6.	Place of Residence			
	Urban	509[25.1]	471[40.6]	981[31]
	Rural	1517[74.9]	689[59.4]	2207[69]
	Total	2027[100]	1161[100]	3188
7.	Sex of Child			
	Male	983[48.5]	615[52.9]	1598[52]
	Female	1044[51.5]	546[47.1]	1590[48]
	Total	2027[100]	1161[100]	3188
8.	Birth Order			
	3-Jan	1058[52.2]	748[64.5]	1807[57]
	6-Apr	639[31.6]	307[26.5]	947[30]
	>7	329[16.2]	105[9.0]	434[13]
	Total	2027[100]	1161[100]	3188
9.	Wealth Index			
	Rich	574[28.3]	618[53.3]	1193{37]
	Middle	359[17.8]	230[19.8]	590[19]
	Poor	1092[53.9]	312[26.9	1405[44]
	Total	2027[100]	1161[100]	3188
10.	Access to Information			
	Yes	913[47.4]	314[28.5]	1227[41]
	No	1011[52.6]	788[71.5]	1799[59]
	Total	1924[100]	1102[100]	3027
11.	Region			
	Islamabad	7[0.4]	7[0.6]	140[0.5]
	Punjab	963[47.5]	802[69.1]	1765[55]
	Sindh	584[28.8]	167[14.4]	752[24]
	KPK	321[15.9]	168[14.5]	490[15]
	Balochistan	132[6.5]	11[1.0]	143[5]
	Gilgit[Baltistan]	17[0.9]	4[0.4]	22[0.5]
	Total	2027[100]	1161[100]	3188
	Place of Delivery			
12	Private hospital	653[32.3]	521[45.0]	1175[37]
	Public Hospital	244[12.1]	231[19.9]	475[15]
	Home	1123[55.6]	408[35.1]	1531[48]
	Total	2020[100]	1161[100]	3182
13.	Use of Antental Care			
	Yes	1378[68.2]	976[84.1]	828[26]
	No	643[31.8]	184[15.9]	2354[74]
	Total	2022[100]	1160[100]	3182
14.	Twin Births			
	Single	2014[99.4]	1151[99.1]	3165[99.3]
	>1	12[0.6]	10[0.9]	22[0.7]
	Total	2027[100]	1161[100]	3188
15.	LHW visit in last 12 months			
	Yes	683[51.7]	635[68.8]	1319[59]
	No	639[48.3]	288[31.2]	928[41]
	Total	1323[100]	924[100]	2248
16.	Visited Health Facility			
	Yes	1676[82.9]	992[85.5]	2669[84]
	No	347[17.1]	168[14.5]	515[16]
	Total	2023[100]	1161[100]	3185
			
17.	Distance From Health Care Delivery			
	Not a big problem	1075[53.2]	872[75.2]	1947[61]
	Big problem	945[46.8]	288[24.8]	1233[39]
	Total	2020[100]	1160[100]	3181

Those respondents who were not visited by LHW during the last 12 months and place of delivery was home had incompletely immunized children. The odds of incomplete immunization were high during bivariate analysis for the following variables: low wealth index (OR=3.77, 95% CI: 2.99-4.74); having illiterate fathers (OR=3.01,95% CI: 2.25-4.03); unemployed fathers (OR=4.70; 95% CI:2.14-10.29); father’s age greater than 35 (OR= 1.18; 95% CI: 0.75-1.87); mother with no formal education (OR=3.81; 95% CI: 2.73-5.33); no access to information (OR=2.26; 95% CI:1.82-2.81); having autonomy in health care decisions; no antenatal care (OR= 2.47; 95% CI:1.92-3.19) multiple pregna (OR=1.04;95% CI:0.30-3.6), age of mother greater than 35 yrs (OR=0.93; 95% CI: 0.70-1.25); born in Baluchistan (OR=3.47,95% CI: 2.21-5.49); rural area dwellers (OR=2.04; 95% CI:1.65-2.51); female gender (OR=1.06; 95% CI: 0.87-1.29); birth order (of last born child) greater than 7 (OR=2.21, 95% CI:1.60-3.06); delivered at home (OR=2.20, 95% CI:1.76-2.74); long distance to health care facility (OR=2.66, 95% CI:2.16-3.28); and no LHW visit in last 12 months (OR=1.91, CI:1.48-2.47).

In final model of regression analysis, we evaluated the association of interest by including all the independent variables. Multicollinearity was assessed between mother’s age and between wealth index and residence, through Pearson correlation, and it was significant at the 0.01 level, so the variables of father’s age and residence were eliminated from the final model. The absence of visit by LHW in last 12 months was the most significant factor when all risk factors were analyzed in last model (Table-II).

**Table-II:** Multinomial Regression Analysis to find the association of Lady Health Worker with immunization.

Multinomial Logistic Egression	LHW	Mother’s Age	Mother’s Education	Father’s Age	Father’s Education	Occupation	Wealth Index	Place of Residence	Region	Place of Delivery	Antenatal Care	Assess O Information	Autonomy in Health Care Decision	Distance from Health Care Facility	Birth Order	Male Gender	Multiple Pregnancy
Model 1	2.06 [1.62,2.63]	0.99 [0.83,1.18]	0.64 [0.57,0.72]														
Model 2	2.17 [1.70,2.77]																
Model 3	2.13 [1.67,2.73]			1.00 [0.82,1.22]	0.91 [0.81,1.04]	0.87 [0.75,1.01]	0.60 [0.52,0.70]										
Model 4	2.13 [1.67,2.72]							0.52 [0.40,0.66]	0.73 [0.65,0.82]								
Model 5	1.99 [1.55,2.56]							0.80 [0.70,0.93]	1.72 [1.23,2.40]	1.63 [1.24,2.14]	1.01 [0.78,1.3]						
Model 6	2.19 [1.71,2.80]														0.63 [0.5,0.75]	0.66 [0.68,0.79]	1.04 [0.3,3.6]
Model 7	1.91 [1.48,2.47]	1.01 [0.84,1.23]	0.76 [0.67,0.87]		0.84 [0.72,0.97]				0.75 [0.66,0.86]	0.87 [0.74,1.01]	1.51 [1.07,2.14]	1.34 [1.01,1.77]	1.06 [0.82,1.37]	0.69 [0.52,0.93]			
P – value	0.0001	0.65	0.001	0.47	0.007	0.51	<0.0001	<0.0001	0.94	<0.0001	<0.0001	<0.0001	0.01	<0.0001	0.02	0.59	0.51

## DISCUSSION

The concept of Lady health workers (LHW) originated from the “Barefoot doctors” of Mao Tse Tung of China.^16^ Hundreds of rural peasants were given basic training and were assigned medical and sanitation duties to overcome the misdistribution of health care facilities. Following the development of the program, the declaration of Alma Ata in September 1978 declared health as a human right.^17^ Community health workers have since provided the community with primary health care, to achieve universal health coverage.

Community health workers have several important duties to perform but vaccinating infants against childhood communicable diseases is one of the most cost-effective public health interventions.^17^ Pakistan has the largest community health worker program in the world that includes more than a 1,00,000 LHWs.^18^ LHWs in Pakistan are playing the most important role in delivering primary health care to mothers and infants and family planning services throughout the country. Every year, thousands of children lost their life to diseases that can be prevented by vaccines. We found that the most significant factor resulting in incomplete immunization of infants was the absence of LHWs in the last 12 months. LHWs serve as the major source of information for mothers, as mothers are more comfortable talking with other women. A study cite that the main source of information among mothers of rural Nigeria on immunizations was health care workers (72.7%).^19^ Our study indicated that LHWs play an important role in decreasing the number of incompletely immunized children. The same idea was supported by a study that showed that the percentage of incompletely immunized children has decreased from 47% in 2001-2002 to 22% in 2008-2009 in part due to the efforts of LHWs.^20^ The program’s success was due to its cost effectiveness, good penetration, high acceptability in community, free interaction with women and households.^21^ However, a study done by Ashlesha and Arnab in 2007 in rural India contradicts this idea by stating that the presence of community health workers in a village was not associated with increase in the immunization coverage.^22^

Reducing child mortality and improving maternal health were two important goals in the Millennium Development Goals (MDGs) set forth by the United Nations in 2000.^22^ Of the approximately 4 million neonatal deaths and half a million maternal deaths worldwide each year, LHWs have contributed in decreasing the infant mortality and maternal mortality rates. In 2006, a study in Punjab province of Pakistan showed that the LHWs contributed to a reduction in infant mortality rate from 250 to 79 per 1, 00,000 live births by health education, family planning and immunization.^23^ In a study done in rural northern India, introduction of a large-scale community-based integrated nutrition and health program reduced neonatal mortality rates in those receiving postnatal home visits by health care workers.^24^

Low maternal education level is an important cause of incomplete immunization of children. Our study showed that children of uneducated mothers were more at risk of being incompletely immunized. A study done in Karachi, Pakistan also showed that mothers’ low educational level was associated with low rates of immunization coverage.^25^ Another study in Nigeria showed that 61.1% of women without any formal education had incompletely immunized their children compared to 13.1% of women with secondary education.^2^ In Uganda, a study showed the percentage of incompletely immunized children decreased with lower maternal education.^27^ On the contrary, in Egypt it was demonstrated that 53.6% of higher-educated mothers did not give vaccination on schedule compared with 50% of illiterate mothers.^28^

Distance from the health facility was also found to be an important variable as people living at long distance from the health facility were less likely to get their children vaccinated. The study of Root et al. supported our results by showing that distance to health services negatively affects local level vaccine efficacy.^29^ However, another study done in Dschang, West Region, Cameroon cites that long distance from the health care facility is only marginally significant (p= 0.05).^30^

Hence, the major risk factor associated with incomplete immunization of children after statistically controlling all other risk factors was absence of Lady Health Worker in the area. Thus strategies should be improved to produce better immunization against preventable diseases.

## CONCLUSION

Visit of LHW in last 12 months was significantly associated with immunization status of children below two years of age in Pakistan. Measures should be taken for immunization by expanding the LHW program to under developed areas around the globe. More focused training, incentives for routine immunization promotion, sustainability of on-going programs and initiation of newer programs will help improve immunization and reduce refusal rates for vaccines globally especially underprivileged areas.
